# Provably Secure and Lightweight Patient Monitoring Protocol for Wireless Body Area Network in IoHT

**DOI:** 10.1155/2023/4845850

**Published:** 2023-02-13

**Authors:** Qi Xie, Dongnan Liu, Zixuan Ding, Xiao Tan, Lidong Han

**Affiliations:** Key Laboratory of Cryptography of Zhejiang Province, Hangzhou Normal University, Hangzhou 311121, China

## Abstract

As one of the important applications of Internet of Health Things (IoHT) technology in the field of healthcare, wireless body area network (WBAN) has been widely used in medical therapy, and it can not only monitor and record physiological information but also transmit the data collected by sensor devices to the server in time. However, due to the unreliability and vulnerability of wireless network communication, as well as the limited storage and computing resources of sensor nodes in WBAN, a lot of authentication protocols for WBAN have been devised. In 2021, Alzahrani et al. designed an anonymous medical monitoring protocol, which uses lightweight cryptographic primitives for WBAN. However, we find that their protocol is defenseless to off-line identity guessing attacks, known-key attacks, and stolen-verifier attacks and has no perfect forward secrecy. Therefore, a patient monitoring protocol for WBAN in IoHT is proposed. We use security proof under the random oracle model (ROM) and automatic verification tool ProVerif to demonstrate that our protocol is secure. According to comparisons with related protocols, our protocol can achieve both high computational efficiency and security.

## 1. Introduction

Wireless body area network (WBAN) exists as a transmission network for body monitoring. It has intellectual network appliances, such as personal wireless terminals, wearable devices, and wireless sensors. Individuals can use network devices to build personalized health networks based on WBAN, and they are substantial participants in the Internet of Health Things (IoHT) application. WBAN is widely used in patient monitoring, physiological parameter measurement, and so on. The measured data are transmitted by the sensor to the devices with a forwarding function in real time using wireless network transmission and then stored in the database of the remote server [1–3]. Using WBAN-based systems, patient-specific electronic medical records can be established, and professionals can analyze medical data through patient electronic records. Moreover, the electronic data of patients can be used for later analysis and diagnosis, and medical personnel can provide targeted medical services based on these data [4].

The communication and interaction of WBAN are based on an open wireless channel, so it is inevitable to face a series of challenges. Attackers can eavesdrop, tamper, intercept publicly transmitted information, and use the obtained information to launch attacks and obtain patients' privacy. This poses a great threat to the medical IoHT and patient privacy [5, 6]. In addition, the WBAN system requires real-time data transmission and timely processing of a large number of communication requests, which makes the energy consumption of infrastructures with limited efficiency very heavy [7]. However, most devices for WBAN have limited computing power, so they cannot perform traditional cryptographic calculations. Moreover, intensive computation will bring about overblown network loads, which will affect the performance of the system. Therefore, the medical field urgently needs a lightweight privacy-protected secure key agreement to meet the above challenges.

In recent years, a lot of anonymous medical key agreements have been proposed. An innovative dynamic ID-based key agreement in telecare medical information system (TMIS) was presented by Chen et al. [8]. However, Xie et al. [9] state that Chen et al.'s scheme cannot defend against off-line password guessing attacks and impersonation attacks and has no privacy protection and perfect forward secrecy. Xie et al. [10] presented a novel authentication protocol for TMIS in 2014, which is considered to be pragmatic and secure. Radhakrishnan and Muniyandi [11] submitted a two-factor key agreement for TMIS based on elliptic curve cryptography (ECC). In 2015, Wang and Zhang [12] solved the anonymity of authentication in WBAN using bilinear pairs, and their scheme could defend against known-key attacks and man-in-middle attacks. However, according to the research of Jiang et al. [13], the protocol cannot resist client forgery attacks, is not suitable for practical applications, and may lead to nonsynchronization of system logs. In 2017, Li et al. [14] proposed an anonymous authentication scheme. It employs lightweight cryptographic primitives (e.g., hash function operations) and asserts that it has realized the mutual authentication of the sensor nodes worn by patients and the hub node and has realized unlinkability and anonymity. Later, Koya et al. [15] stated that it is not feasible because their scheme assumes that the central node is entirely credible. Moreover, it is defenseless to sensor impersonation attacks. Soni and Singh [16] submitted a lightweight authentication scheme employing low-cost operations for WBAN. Based on the wireless medical sensor network, Jan et al. [17] submitted a patient key agreement for the healthcare system to realize secure and efficient communication between users and sensors. Recently, Ullah et al. [18] submitted a hyperelliptic curve and pragmatic IoT-based crossdomain authentication scheme for WBAN. In addition, Ullah et al. [19–21] proposed a multimessage signcryption protocol, anonymous certificateless signcryption protocol, and certificate-founded signcryption protocol for IoHT. Khan et al. [22] proposed an online-offline certificate-less signature protocol for IoHT.

Wu et al. [23] designed an identity authentication scheme using unilateral bilinear pairing technology which only performs bilinear pairing at the access point (AP). After that, Chen and Peng [24] declared that it cannot realize mutual authentication and is also susceptible to client forgery attacks. Li et al. [25] devised a key agreement founded on ECC to realize user anonymity. But Sowjanya et al. [26] found that their scheme not only has the problems of clock nonsynchronization and excessive control power of users but also no perfect forward secrecy. Kalra and Sood [27] submitted a secure key agreement that is not affected by time synchronization, which is based on the password. In 2021, Chunka et al. [28] reviewed their scheme and found that it had many security issues. For instance, due to the defects in the gateway design, the scheme cannot confirm the authenticities of sensor nodes, so it cannot resist the sensor nodes captured attacks, and the gateway private key is prone to be leaked. In addition, a large number of redundant multiple hash calculations increase the computational burden on the system. Xu et al. [29] raised an anonymous and lightweight patient monitoring protocol using lightweight cryptographic primitives. The survey of Alzahrani et al. [30] shows that off-line identity guessing attacks will wreck its anonymity, and it is also defenseless to key compromise attacks and replay attacks.

### 1.1. Motivation and Contributions

According to the summary of the existing literature [30–33], we found that some protocols using lightweight cryptographic primitives cannot resist various attacks, and many protocols based on asymmetric cryptography have high time complexity. In 2021, Alzahrani et al. [30] designed an anonymous medical monitoring scheme. Nevertheless, their scheme is defenseless to stolen-verifier attacks, known-key attacks, and off-line identity guessing attacks and has no perfect forward secrecy. To realize a secure and lightweight authentication protocol in WBAN systems, we propose a patient monitoring protocol. Here, our contributions are as follows:

- We reviewed Alzahrani et al.'s [30] protocol and analyzed its drawbacks, for example, known-key attacks, stolen-verifier attacks, and off-line identity guessing attacks
- A patient monitoring protocol is proposed to realize the security and lightweight requirements of WBAN systems
- Using the automated verification tool ProVerif and formal security proof in ROM, we demonstrate the proposed protocol is secure
- Our protocol is relatively pragmatic and secure by performance comparison

The remaining section is constructed as follows: the system model and preliminaries are given in Section 2. In Section 3, we describe the review and drawbacks of Alzahrani et al.'s protocol.  Section 4 proposes a patient monitoring scheme. Its security is analyzed in Sections 5 and 6. Its security properties, computation cost, storage cost, and communication cost between ours and some related protocols are evaluated in Section 7.  Section 8 concludes the paper.

## 2. System Model and Preliminaries

In this section, we present the system model and attack model. Concurrently, we describe the physically unclonable function (PUF).

### 2.1. System Model

Figure 1 illustrates its system model. It adopts the centralized two-hop architecture of WBAN, which includes the following devices: sensor nodes (SNs), relay nodes (RNs), and medical server node (MS). RN is the intermediate node, and only needs to forward messages between SN and MS, and it can add or delete its identity before forwarding messages. RN is always within the communication coverage of MS, and SN is covered by at least one RN. Resource-constrained SN monitors and collects patients' medical health data by being worn or embedded into patients.

### 2.2. Attack Model

Presuming the attacker (AR) maintains the following capacities:

1. AR can capture messages transmitted via open channels and may eavesdrop, replace, replay, or intercept the data in these messages
2. AR can obtain verifier table stored in MS, but cannot obtain its secret key
3. AR can capture *SN*_*j*_ and RN and then retrieve all data stored in their memory
4. We adopt Dolev–Yao threat model [34] and assume that the public channel is insecure

### 2.3. Physically Unclonable Function

As a hardware security technology, a physically unclonable function (PUF) can be regarded as the “digital fingerprint” of the chip [35]. It uses the inherent physical differences to produce a specific unclonable response to a given challenge. Therefore, it is difficult to be predicted before production and cloned after production. It has broad application prospects in the field of security. According to the same challenge, the response of PUF can remain unchanged under different conditions. Any detection or observation of PUF will change the circuit characteristics, and the output of PUF will also change. Therefore, PUF is often used to protect crucial data in cryptography [36].

All notations in our paper are illustrated in Table 1.

## 3. Drawbacks of Alzahrani et al.'s Scheme

### 3.1. Review of Alzahrani et al.'s Scheme

We briefly review Alzahrani et al.'s [30] anonymous authentication protocol, which involves three steps: (1) system initialization; (2) device registration; (3) mutual authentication and key agreement. SA performs step (1) and step (2) through a private channel as follows.

#### 3.1.1. System Initialization

- SA generates a long-term master secret key *K*_*MS*_ for MS
- Subsequently, MS reserves the master secret key *K*_*MS*_

#### 3.1.2. Devices Registration

- SA selects three random integers *r*, *P*_*R*1_, *P*_*R*2_, and an identity *id*_*j*_ for the sensor node *SN*_*j*_ and reserves tuple <*id*_*j*_, *P*_*R*1_, *P*_*R*2_> in the memory of MS
- SA computes *x*_*N*__*j*_=*r* ⊕ *K*_*MS*_, *y*_*N*__*j*_ =  *id*_*j*_⊕*h*(*K*_*MS*_, *r*)
- SA reserves tuple <*id*_*j*_, *x*_*N*__*j*_, *y*_*N*__*j*_, *P*_*R*1_, *P*_*R*2_> in the memory of *SN*_*j*_
- Finally, the verification table of MS is <*id*_*j*_, *P*_*R*1_, *P*_*R*2_, *id*_*R*_>

#### 3.1.3. Mutual Authentication and Key Agreement

The communications between *SN*_*j*_ and MS are as follows:

- *SN*_*j*_ creates a current timestamp *T*_1_ and computes the validation *Vid*_*j*_=*h*(*id*_*j*_, *x*_*N*__*j*_, *y*_*N*__*j*_, *P*_*R*2_, *T*_1_), where *id*_*j*_ is *SN*_*j*_'s identity, *x*_*N*__*j*_=*r* ⊕ *K*_*MS*_, *y*_*N*__*j*_=*id*_*j*_ ⊕ *h*(*K*_*MS*_, *r*), *P*_*R*2_ denotes a random integer, and the current timestamp is denoted as *T*_1_.
- *SN*_*j*_ submits Message1 tuple <*x*_*N*__*j*_, *y*_*N*__*j*_, *Vid*_*j*_, *T*_1_> to RN.
- RN appends its identity *id*_*R*_ and forwards the Message2 tuple <*x*_*N*__*j*_, *y*_*N*__*j*_, *Vid*_*j*_, *T*_1_, *id*_*R*_> to MS.
- MS scans the identity *id*_*R*_ and finishes the session if no record is found in its memory. Otherwise, MS creates the current timestamp *T*_2_ and checks if |*T*_2_ − *T*_1_| ≤ Δ*T*, and if not, finishes the session. Otherwise, MS computes *r*^*∗*^=*x*_*N*__*j*_ ⊕ *K*_*MS*_, *id*_*j*_^*∗*^=*y*_*N*__*j*_ ⊕ *h*(*K*_*MS*_, *r*^*∗*^). MS checks the validity of the identity *id*_*j*_^*∗*^, if so, MS extracts the tuple <*id*_*j*_^*∗*^, *P*_*R*1_, *P*_*R*2_> from its memory, computes *Vid*_*j*_^*∗*^=*h*(*id*_*j*_^*∗*^, *x*_*N*__*j*_, *y*_*N*__*j*_, *P*_*R*2_, *T*_1_), and checks *Vid*_*j*_^*∗*^ ? *=* *Vid*_*j*_. If so, MS generates random nonce *m* and *r*^new^ and computes *s*=*id*_*j*_^*∗*^ ⊕ *y*_*N*__*j*_, *j*=*id*_*j*_^*∗*^ ⊕ *x*_*N*__*j*_, *v*=*m* ⊕ *s*, *x*_*N*__*j*_^new^=*r*^new^ ⊕ *K*_*MS*_, *y*_*N*__*j*_^new^=*id*_*j*_^*∗*^ ⊕ *h*(*K*_*MS*_, *r*^new^), *g*=*h*(*m*, *s*, *j*, *P*_*R*2_), *u*=*x*_*N*__*j*_^new^ ⊕ *g*, *n*=*y*_*N*__*j*_^new^ ⊕ *g*, Δ=*h*(*m*, *id*_*j*_^*∗*^, *s*, *x*_*N*__*j*_^new^, *y*_*N*__*j*_^new^), and the session key *K*_*SH*_=*h*(*m*, *j*, *P*_*R*1_, *P*_*R*2_). Afterwards, MS sends the Message3 tuple <*v*, *u*, Δ, *n*, *id*_*R*_> to RN. MS displaces *P*_*R*1_ with *P*_*R*2_ and *P*_*R*2_ with *K*_*SH*_.
- RN removes its identity *id*_*R*_ and forwards the Message 4 tuple <*v*, *u*, Δ, *n*> to *SN*_*j*_.
- *SN*_*j*_ computes *s*^*∗*^=*id*_*j*_ ⊕ *y*_*N*__*j*_, *m*^*∗*^=*v* ⊕ *s*^*∗*^, *j*^*∗*^=*id*_*j*_ ⊕ *x*_*N*__*j*_, *g*^*∗*^=*h*(*m*^*∗*^, *s*^*∗*^, *j*^*∗*^ *P*_*R*2_), *x*_*N*__*j*_^new+^=*u* ⊕ *g*^*∗*^, *y*_*N*__*j*_^new+^=*n* ⊕ *g*^*∗*^, Δ^*∗*^=*h*(*m*^*∗*^, *id*_*j*_, *s*^*∗*^, *x*_*N*__*j*_^new+^, *y*_*N*__*j*_^new+^). Afterwards, *SN*_*j*_ checks Δ^*∗*^ ?=Δ. If so, *SN*_*j*_ computes the session key *K*_*SH*_=*h*(*m*^*∗*^, *j*^*∗*^, *P*_*R*1_, *P*_*R*2_). *SN*_*j*_ displaces *x*_*N*__*j*_ and *y*_*N*__*j*_, with *x*_*N*__*j*_^new+^ and *y*_*N*__*j*_^new+^, and stores them in its memory. Finally, *SN*_*j*_ displaces *P*_*R*1_ with *P*_*R*2_ and *P*_*R*2_ with *K*_*SH*_.

### 3.2. Drawbacks

#### 3.2.1. Off-Line Identity Guessing Attack

Supposing an adversary (AR) can eavesdrop on the conversation between *SN*_*j*_ and MS. AR intercepts the first round of *x*_*N*__*j*−1_, *y*_*N*__*j*−1_, and the second round of *x*_*N*__*j*−2_, *y*_*N*__*j*−2_, where *x*_*N*__*j*−2_ and *y*_*N*__*j*−2_ are the first round of *x*_*N*__*j*−1_^new+^ and *y*_*N*__*j*−1_^new+^. AR computes Δ^*∗*^=*h*(*m*^*∗*^, *id*_*j*_, *s*^*∗*^, *x*_*N*__*j*−1_^new+^, *y*_*N*__*j*−1_^new+^), where *m*^*∗*^=*v* ⊕ *s*^*∗*^, *s*^*∗*^=*id*_*j*_ ⊕ *y*_*N*__*j*_. Only *id*_*j*_ in Δ^*∗*^ is unknown, and AR guesses *id*_*j*_ to verify if Δ^*∗*^ ? *=* Δ. If so, AR obtains *id*_*j*_ successfully. Otherwise, guesses *id*_*j*_ again.

#### 3.2.2. Desynchronization Attack

If AR intercepts Message4 and drops it, the *SN*_*j*_ will miss it. The insecurity is that MS has updated *x*_*N*__*j*_, *y*_*N*__*j*_, *P*_*R*1_, *P*_*R*2_, but *SN*_*j*_ has not. This will make every subsequent authentication process between *SN*_*j*_ and MS fail.

#### 3.2.3. Stolen-Verifier Attack

If the verifier table <*id*_*j*_, *P*_*R*1_, *P*_*R*2_, *id*_*R*_> of MS is stolen, AR can obtain all the data in it. AR eavesdrops on the communication between *SN*_*j*_ and MS, intercepts Message1 tuple <*x*_*N*__*j*_, *y*_*N*__*j*_, *Vid*_*j*_, *T*_1_>, Message 4 tuple <*v*, *u*, Δ, *n*>, computes *s*^*∗*^=*id*_*j*_ ⊕ *y*_*N*__*j*_, *m*^*∗*^=*v* ⊕ *s*^*∗*^, and *j*^*∗*^=*id*_*j*_ ⊕ *x*_*N*__*j*_, and computes the session key *K*_*SH*_=*h*(*m*^*∗*^, *j*^*∗*^, *P*_*R*1_, *P*_*R*2_). That is, AR can obtain the session key.

#### 3.2.4. Known-Key Attack

If the session keys of two consecutive rounds are leaked, AR will get *P*_*R*1−3_ and *P*_*R*2−3_ of the third round. According to identity guessing attacks, AR obtains the SN's identity *id*_*j*_. In the third round of protocol execution, AR intercepts message 1 and message 4 and computes *s*^*∗*^=*id*_*j*_ ⊕ *y*_*N*__*j*−3_, *m*^*∗*^=*v* ⊕ *s*^*∗*^, *g*^*∗*^=*h*(*m*^*∗*^, *s*^*∗*^, *j*^*∗*^ *P*_*R*2−3_), *x*_*N*__*j*−3_^new+^=*u* ⊕ *g*^*∗*^, *y*_*N*__*j*−3_^new+^=*n* ⊕ *g*^*∗*^, *K*_*SH*_=*h*(*m*^*∗*^, *j*^*∗*^, *P*_*R*1−3_, *P*_*R*2−3_). Therefore, the session key of the subsequent round will be obtained by the AR.

#### 3.2.5. No Perfect Forward Security

If the long-term secret key *K*_*MS*_ and short-term secret key *P*_*R*1_ and *P*_*R*2_ of the Alzahrani et al.'s [30] scheme are leaked, AR calculates *r*^*∗*^=*x*_*N*__*j*_ ⊕ *K*_*MS*_, *id*_*j*_=*y*_*N*__*j*_ ⊕ *h*(*K*_*MS*_, *r*^*∗*^). Then, AR calculates *s*^*∗*^=*id*_*j*_ ⊕ *y*_*N*__*j*_, *m*^*∗*^=*v* ⊕ *s*^*∗*^, *g*^*∗*^=*h*(*m*^*∗*^, *s*^*∗*^, *j*^*∗*^, *P*_*R*2_). Finally, AR can compute the session key *K*_*SH*_=*h*(*m*^*∗*^, *j*^*∗*^, *P*_*R*1_, *P*_*R*2_). Therefore, it doesn't achieve perfect forward secrecy.

## 4. Proposed Protocol

A security-enhanced protocol is presented, which involves three steps: (1) system initialization; (2) device registration; (3) mutual authentication and key agreement. SA executes initialization and registration steps through a private channel as follows.

### 4.1. Initialization

SA executes as follows:

1. The master secret key *K*_*MS*_ is generated by SA
2. Subsequently, MS accepts the master secret key *K*_*MS*_ via a secure channel and keeps it secretly
3. SA chooses an elliptic curve *E*_*c*_(*α*, *β*) of large order. *P* is a base point. SA computes *Q*=*K*_*MS*_∙*P*. Afterwards, SA chooses a hash function *h*(∙).

### 4.2. Registration

The registration phase can be described as follows:

1. SA chooses the random integer *a*_*j*_ and the identity *id*_*j*_ for the sensor node *SN*_*j*_, an identity *id*_*R*_ for RN, and reserves *id*_*j*_ and *id*_*R*_ in the memory of MS
2. SA computes *x*_*N*__*j*_=*a*_*j*_ ⊕ *h*(*K*_*MS*_, *T*_*j*_), *y*_*N*__*j*_=*id*_*j*_ ⊕ *h*(*K*_*MS*_, *a*_*j*_, *T*_*j*_), *MH*_*j*_=*h*(*id*_*j*_, *K*_*MS*_), where *T*_*j*_ is the current timestamp, and *K*_*MS*_ is MS's secret key
3. SA reserves the tuple <*id*_*j*_, *x*_*N*__*j*_, *y*_*N*__*j*_, *MH*_*j*_, *T*_*j*_> in the memory of *SN*_*j*_, and *SN*_*j*_ generates a challenge Cha_*j*_ and computes Res_*j*_=PUF(Cha_*j*_), *ST*_*j*_=*h*(Res_j_)  ⊕  *MH*_*j*_, where PUF is deployed in the sensor node *SN*_*j*_
4. Finally, *SN*_*j*_ stores {*id*_*j*_, *x*_*N*__*j*_, *y*_*N*__*j*_, ST_j_, Cha_j_, T_j_}, and the verification table of MS is {*id*_*R*_, *id*_*j*_}

### 4.3. Mutual Authentication and Key Agreement

This phase is shown in Figure 2.

1. *SN*_*j*_ chooses the random integer *b*_*j*_ and the timestamp *T*_1_ and calculates *MH*_*j*_=*h*(PUF(Cha_*j*_)) ⊕ *ST*_*j*_, *A*_1_=*b*_*j*_∙*P*, *A*_2_=*b*_*j*_∙*Q*, *Vid*_*j*_=*h*(*id*_*j*_, *x*_*N*__*j*_, *y*_*N*__*j*_, *A*_1_, *A*_2_, *h*(*A*_2_, *MH*_*j*_), *T*_*j*_, *T*_1_).
2. *SN*_*j*_ submits the Message1 tuple <*x*_*N*__*j*_, *y*_*N*__*j*_, *Vid*_*j*_, *A*_1_, *T*_*j*_, *T*_1_> to RN.
3. RN appends its identity *id*_*R*_ and forwards the Message 2 tuple <*x*_*N*__*j*_, *y*_*N*__*j*_, *Vid*_*j*_, *A*_1_, *T*_*j*_, *T*_1_, *id*_*R*_> to MS.
4. MS scans the identity *id*_*R*_ and finishes the session if no record is found in its memory. Otherwise, MS creates the current timestamp *T*_2_ and checks if |*T*_2_ − *T*_1_| ≤ Δ*T*, and if not, finishes the session. Otherwise, MS computes *a*_*j*_=*x*_*N*__*j*_ ⊕ *h*(*K*_*MS*_, *T*_*j*_), *id*_*j*_^*∗*^=*x*_*N*__*j*_ ⊕ *h*(*K*_*MS*_, *a*_*j*_, *T*_*j*_). MS calculates *A*_2_^*∗*^=*K*_*MS*_∙*A*_1_, *Vid*_*j*_^*∗*^=*h*(*id*_*j*_^*∗*^, *x*_*N*__*j*_, *y*_*N*__*j*_, *A*_1_, *A*_2_^*∗*^, *h*(*A*_2_^*∗*^, *h*(*id*_*j*_^*∗*^, *K*_*MS*_)), *T*_*j*_, *T*_1_) and checks *Vid*_*j*_^*∗*^*?* *=* *Vid*_*j*_. If so, MS creates random numbers *a*_*i*_ and *b*_*i*_. Next, MS computes *A*_3_=*b*_*i*_∙*P*, *A*_4_=*b*_*i*_∙*A*_1_, *x*_*N*__*j*_^new^=*a*_*i*_ ⊕ *h*(*K*_*MS*_, *T*_2_), *y*_*N*__*j*_^new^=*id*_*j*_^*∗*^ ⊕ *h*(*K*_*MS*_, *a*_*i*_, *T*_2_), *μ*=*x*_*N*__*j*_^new^ ⊕ *h*(*A*_2_^*∗*^, *h*(*id*_*j*_^*∗*^, *K*_*MS*_), *T*_2_), *λ*=*y*_*N*__*j*_^new^ ⊕ *h*(*T*_2_, *A*_2_^*∗*^, *h*(*id*_*j*_^*∗*^, *K*_*MS*_)), the session key *K*_*SH*_=*h*(*A*_1_, *A*_2_^*∗*^, *A*_3_, *A*_4_, *id*_*j*_^*∗*^, *T*_2_), and Δ=*h*(*x*_*N*__*j*_^new^, *y*_*N*__*j*_^new^, *K*_*SH*_, *T*_2_). Afterwards, MS sends the Message3 tuple <*μ*, *λ*, Δ, *A*_3_, *T*_2_, *id*_*R*_> to RN.
5. RN removes its identity *id*_*R*_ and forwards the Message4 tuple <*μ*, *λ*, Δ, *A*_3_, *T*_2_> to *SN*_*j*_.
6. *SN*_*j*_ creates the current timestamp *T*_3_ and checks if |*T*_3_ − *T*_2_| ≤ Δ*T*, and if not, finishes the session. Otherwise, *SN*_*j*_ computes *A*_4_^*∗*^=*b*_*j*_∙*A*_3_, *x*_*N*__*j*_^new*∗*^=*μ* ⊕ *h*(*A*_2_, *MH*_*j*_, *T*_2_), *y*_*N*__*j*_^new*∗*^=*λ* ⊕ *h*(*T*_2_, *A*_2_, *MH*_*j*_), *K*_*SH*_=*h*(*A*_1_, *A*_2_, *A*_3_, *A*_4_^*∗*^, *id*_*j*_, *T*_2_), Δ^*∗*^=*h*(*x*_*N*__*j*_^new*∗*^, *y*_*N*__*j*_^new*∗*^, *K*_*SH*_, *T*_2_). *SN*_*j*_ checks if Δ^*∗*^ ? *=* Δ. If so, *SN*_*j*_ successfully establishes the session key *K*_*SH*_ with MS and updates <*x*_*N*__*j*_, *y*_*N*__*j*_, T_j_> with <*x*_*N*__*j*_^new*∗*^, *y*_*N*__*j*_^new*∗*^, *T*_2_>.

## 5. Informal Security Analysis

### 5.1. Off-Line Identity Guessing Attack

If an adversary(AR) can eavesdrop on the open channel and guess *id*_*j*_ of the sensor node SN_j_, it is not feasible for him/her to verify whether *Vid*_*j*_^*∗*^ ? *=* *Vid*_*j*_ is correct or not without knowing *A*_2_, where *A*_2_ = *b*_*j*_∙*K*_*MS*_∙*P*, *Vid*_*j*_=*h*(*id*_*j*_, *x*_*N*__*j*_, *y*_*N*__*j*_, *A*_1_, *A*_2_, *h*(*A*_2_, *MH*_*j*_), *T*_*j*_, *T*_1_), *MH*_*j*_=*h*(*id*_*j*_, *K*_*MS*_). Because of computational Diffie–Hellman problem (CDHP), AR cannot compute *A*_2_=*b*_*j*_∙*K*_*MS*_∙*P* from *A*_1_=*b*_*j*_∙*P* and *Q*=*K*_*MS*_∙*P*. Therefore, off-line identity guessing attack is infeasible.

### 5.2. Desynchronization Attack

In the improved protocol, *x*_*N*__*j*_ and *y*_*N*__*j*_ are updated as *x*_*N*__*j*_^new^ and *y*_*N*__*j*_^new^ on the side of the MS. Even if AR intercepts the Message4, it has no impact on the next session between the sensor node *SN*_*j*_ and the MS.

### 5.3. Stolen-Verifier Attack

Stolen-verifier attack means that an adversary can obtain verification table except the secret key from MS by trespassing on the device or side channel attack and then launch attacks. In the proposed scheme, the verification table of MS only contains the identities *id*_*j*_ and *id*_*R*_ of *SN*_*j*_ and *RN*. So the adversary cannot launch any attacks even if he or she obtains these identities. Thus, the protocol defends against stolen-verifier attacks.

### 5.4. Known-Key Attack

Assuming that AR knows the session key *K*_*SH*_=*h*(*A*_1_, *A*_2_, *A*_3_, *A*_4_^*∗*^, *id*_*j*_, *T*_2_), because *K*_*SH*_ only contained in Δ^*∗*^=*h*(*x*_*N*__*j*_^new*∗*^, *y*_*N*__*j*_^new*∗*^, *K*_*SH*_, *T*_2_), so AR cannot launch any attack.

### 5.5. Smart Card Lost Attack

By the side-channel attack, AR is able to get all data reserved in the smart card when it is lost, and then launch attacks. However, in our protocol, smart card isn't used, so the protocol defends against the smart card lost attack.

### 5.6. Sensor Node Captured Attack

In the improved protocol, the sensor node *SN*_*j*_ stores {*id*_*j*_, *x*_*N*__*j*_, *y*_*N*__*j*_, *ST*_*j*_, Cha_*j*_, *T*_*j*_}, where *id*_*j*_ is *SN*_1_'s identity, *x*_*N*__*j*_=*a*_*j*_ ⊕ *h*(*K*_*MS*_, *T*_*j*_), *y*_*N*__*j*_ ⊕ *id*_*j*_ ⊕  *h*(*K*_*MS*_, *a*_*j*_, *T*_*j*_), *ST*_*j*_=*h*(PUF(Cha_*j*_)) ⊕ *MH*_*j*_, Cha_*j*_ is the challenge of PUF(), *T*_*j*_ is the timestamp, and *K*_*MS*_ is the secret key of MS. Assuming that the sensor node *SN*_*j*_ is captured by AR, he/she cannot obtain the secret parameter *MH*_*j*_ to impersonate *SN*_*j*_ because of PUF. In addition, AR cannot obtain the secret key *K*_*MS*_. Therefore, the sensor node captured attack cannot influence the security of nodes and the sensor network.

### 5.7. Anonymity and Unlinkability

The identity *id*_*j*_ of the sensor node *SN*_*j*_ is in Message 1={*x*_*N*__*j*_, *y*_*N*__*j*_, *Vid*_*j*_, *A*_1_, *T*_*j*_, *T*_1_} and transmitted via an open channel, where *Vid*_*j*_=*h*(*id*_*j*_, *x*_*N*__*j*_, *y*_*N*__*j*_, *A*_1_, *A*_2_, *h*(*A*_2_, *MH*_*j*_)*T*_*j*_, *T*_1_), *MH*_*j*_=*h*(*id*_*j*_, *K*_*MS*_), *y*_*N*__*j*_=*id*_*j*_ ⊕  *h*(*K*_*MS*_, *a*_*j*_, *T*_*j*_). So an adversary cannot compute the identity *id*_*j*_ of the sensor *SN*_*j*_ because he can not know the secret key *K*_*MS*_ of MS. Thus, our scheme achieves anonymity. Moreover, because each session will generate new *b*_*j*_ and *T*_*j*_, the identity *id*_*j*_ of the sensor node *SN*_*j*_ cannot be tracked by AR.

### 5.8. Perfect Forward Secrecy

If AR obtains all the secret information of the sensor node *SN*_*j*_ and the long-term master secret key *K*_*MS*_ of MS, because of CDHP, he/she still cannot successfully calculate *K*_*SH*_=*h*(*A*_1_, *A*_2_, *A*_3_, *A*_4_^*∗*^, *id*_*j*_, *T*_2_) without knowing *A*_4_^*∗*^. Therefore, the protocol achieves perfect forward secrecy.

### 5.9. Impersonation Attack

This attack means that AR can impersonate a legal user to generate and send a message, and the message can be passed through the authentication by the receiver. That is to say, the receiver confirms that the message is initiated by a legitimate user. In our protocol, AR impersonates the sensor node *SN*_*j*_ to generate and send {*x*_*N*__*j*_, *y*_*N*__*j*_, *Vid*_*j*_, *A*_1_, *T*_*j*_, *T*_1_} to RN, where *x*_*N*__*j*_=*a*_*j*_ ⊕  *h*(*K*_*MS*_, *T*_*j*_), *y*_*N*__*j*_=*id*_*j*_ ⊕  *h*(*K*_*MS*_, *a*_*j*_, *T*_*j*_), *Vid*_*j*_=*h*(*id*_*j*_, *x*_*N*__*j*_, *y*_*N*__*j*_, *A*_1_, *A*_2_, *h*(*A*_2_, *MH*_*j*_)*T*_*j*_, *T*_1_), *K*_*MS*_ is MS's secret key, and *T*_1_ is the timestamp. The adversary cannot forge *x*_*N*__*j*_ and *y*_*N*__*j*_ without knowing *K*_*MS*_. On the other hand, the adversary cannot compute *MH*_*j*_ even if he/she can obtain all data stored in *MH*_*j*_ due to the property of PUF. Therefore, the adversary cannot generate the valid *Vid*_*j*_.

### 5.10. Replay Attack

If AR can obtain a message and replay it to the receiver, the message can be passed through the authentication of the receiver. In the proposed scheme, the timestamps and random nonce are used, so the protocol defends against the replay attack.

## 6. Formal Security Analysis

### 6.1. Formal Verification Using ProVerif

As an automated verification cryptographic scheme tool, ProVerif [37] is founded on the Dolev–Yao model and Prolog language. It verifies many cryptographic primitives, for example, public-key cryptography, hash function, and equations. When using ProVerif tool for verifying insecure cryptographic protocols, the tool will give a corresponding attack sequence.

The open channel, types, constants, variables, constructors, and destructors of our proposed protocol are represented in Figure 3. We designed four events for the improved protocol, which are BeginSNj(), BeginMS(), EndSNj(), and EndMS() as depicted in Figure 4. BeginSNj() represents that the sensor node *SN*_*j*_ begins the key agreement session with MS. BeginMS() represents that MS starts the key agreement session with *SN*_*j*_. *SN*_*j*_ successfully established a session key with MS, which is indicated as EndSNj(). EndMS() represents MS successfully established a session key with the sensor node *SN*_*j*_.

Queries are shown in Figure 5. Figures 6 and 7 are exhibiting the processes of the sensor node SN_j_ and MS. The main process is represented in Figure 8.

For testifying the improved scheme's correctness, we propose some queries and finally implement them through simulation, as shown in Figure 9.

Results (1)–(4) proved that the secret parameters and session key are secure, and sensor nodes are anonymous in our protocol. Results (5)-(7) showed that the two processes began and terminated successfully in sequence.

### 6.2. Formal Security Proof

After identifying the random oracle model (ROM), we calculate the advantage of breaking our protocol *𝒫* by the adversary *A*. The notions of ROM are clarified as follows.

#### 6.2.1. Participants & States

Three participants *P* is in *𝒫*, sensor node *SN*, relay node *RN*, and medical server node *MS*. In *i-th* instance, *P*, *SN*, *RN*, and *MS* are recorded as INS_*P*_^*i*^, INS_*SN*_^*i*^, INS_*RN*_^*i*^, and INS_*MS*_^*i*^, respectively. The oracles in ROM have only three states: Accept, Reject, and ⊥. Accept represents a correct message that is received by an oracle. If the message is illegal, the oracle in Reject. ⊥ means both the conditions above have not occurred.

If the oracle INS_*SN*_^*i*^(INS_*MS*_^*i*^) is in Accept, and the session key *K*_*SN*_^*i*^(*K*_*MS*_^*i*^) has been agreed with INS_*MS*_^*i*^(INS_*SN*_^*i*^), then INS_*SN*_^*i*^(INS_*MS*_^*i*^) gets the session identity SID_*SN*_^*i*^(SID_*MS*_^*i*^), and its participant's identity is PID_*SN*_^*i*^(PID_*MS*_^*i*^).

#### 6.2.2. Partnering

If INS_*SN*_^*i*^ and INS_*MS*_^*i*^ are in Accept, the session key is negotiated. Two partners meet below requirements:

1. *K*_*SN*_^*i*^=*K*_*MS*_^*i*^
2. SID_*SN*_^*i*^=SID_*MS*_^*i*^
3. PID_*SN*_^*i*^=INS_*MS*_^*i*^, PID_*MS*_^*i*^=INS_*SN*_^*i*^

#### 6.2.3. Queries

Queries can emulate multiple attacks.

 
*Execute*(INS_*P*_^*i*^)if the query is lunched by *A*, he/she gets all the transcripts.
 
*Send* (INS_*P*_^*i*^*, Message*): which simulates that *Message* is sent to INS_*P*_^*i*^. If the message is correct, INS_*P*_^*i*^ responses *A*, else, the message is ignored.
 
*Reveal*(INS_*SN*_^*i*^, INS_*MS*_^*i*^)if INS_*SN*_^*i*^ and INS_*MS*_^*i*^ are in the state Accept, the session key has been agreed, and the query *Test* has not been executed yet. Then, the session key will be revealed by this query. Else, return null.
 
*Corrupt*(INS_*SN*_^*i*^)which simulates the attack of intercepting *SN*_*j*_ and returns the stored information {*id*_*j*_, *x*_*N*__*j*_, *y*_*N*__*j*_, *ST*_*j*_, Cha_*j*_, PUF(), *T*_*j*_} in it.
 
*Test*(INS_*SN*_^*i*^)this query produces a random bit *r*, which is performed no more than once. If *r*=1 and the session key has been agreed, the real session key is returned to *A*, else, the query returns a random session key.

#### 6.2.4. Freshness

If the ensuing requirements are met, INS_*P*_^*i*^ can be defined as fresh.

1. INS_*SN*_^*i*^ and INS_*MS*_^*i*^ are in the state Accept
2. Reveal has not been executed
3. Corrupt is executed at most once

#### 6.2.5. Semantic Security

The random bit *r* in *Test* query determines the output of *Test*. Meanwhile, *A* generates a random *r*′, if *r*′=*r*, *A* knows if the output is session key. The advantage of guessing the correct bit is Adv_*𝒫*_^*A*^=|2 Pr [*r*=*r*′] − 1|=|2 Pr [suc(*A*)] − 1|. *𝒫* is secure when Adv_*𝒫*_^*A*^ < *η*, where *η* is sufficiently small.

CDHP: the CDHP is specified that given *P*, *aP*, and *bP*, computing *abP* is computationally infeasible in probabilistic polynomial time (PPT). *P* is the generator point, *a*, *b* ∈ *Z*_*p*_. Subsequently, the advantage of solving CDHP is Adv_*A*_^CDHP^=Pr   [*A*(*P*, *aP*, *bP*)=*abP* : *P* ∈ *E*(*F*_*p*_); *a*, *b* ∈ *Z*_*p*_], Adv_*A*_^CDHP^ < *η*.

**Theorem 1 .**

Suppose the adversary *A* tends to break the proposed scheme *𝒫* in PPT. The queries Execute, Send, and Hash are executed *q*_*E*_, *q*_*S*_, and *q*_*H*_ times, respectively. Query Test is allowed to be executed at most once. *l*_*h*_ is the bit-length of the hash operation's the output. *n*=2^*l*_*t*_^, where *l*_*t*_ is the average length of other transcripts. The advantage of breaking *𝒫* by *A* in PPT can be expressed as follows:

(1) $$\begin{array}{c} Adv_{A}^{P}\leq \frac{{\left(q_{S}+q_{E}\right)}^{2}}{n}+\frac{q_{H}^{2}}{2^{l_{h}}}+2Adv_{A}^{CDHP}+2Adv_{A}^{PUF}\text{.} \end{array}$$

**Proof**

To simulate the attacks on *𝒫*, we define various games Game_*i*_(0 < *i* < 3). The event Success_*A*_^*i*^(0 < *i* < 3) corresponding to Game_*i*_ means that *A* completes his/her goal in Game_*i*_.

Game_0_: which simulates the real attack, at the first, the probability of *A* cracking *𝒫* is
  (2) $$\begin{array}{c} \begin{array}{c} Adv_{A}^{P}=\left|2\;\mathrm{Pr}\;\left[Success_{A}^{0}\right]-1\right| \end{array}\text{.} \end{array}$$
Game_1_: which simulates that *A* launches *Execute* and *Test* queries to verify the output according to the transcripts {Message1, Message2, Message3, Message4}. Among the transcripts, {*A*_1_, Δ, *A*_3_, *T*_2_} are related to the session key. However, *A* cannot figure out the relation between them the transcripts and the output of *Test* because of the random numbers. Therefore, we have
  (3) $$\begin{array}{c} \mathrm{Pr}\;\left[Success_{A}^{1}\right]=\mathrm{Pr}\;\left[Success_{A}^{0}\right]. \end{array}$$
Game_2_: In this game, we simulate *A* computes the session key *K*_*SH*_ through the messages transmitted openly. *K*_*SH*_=*h*(*A*_1_, *A*_2_^*∗*^, *A*_3_, *A*_4_, *id*_*j*_^*∗*^, *T*_2_), which is based on CDHP. The advantage of calculating *K*_*SH*_ by *A* is Adv_*A*_^CDHP^. Therefore, we have
  (4) $$\begin{array}{c} \mathrm{Pr}\;\left[Success_{A}^{2}\right]-\mathrm{Pr}\;\left[Success_{A}^{1}\right]=Adv_{A}^{CDHP}\text{.} \end{array}$$
Game_3_: This game simulates *A* performs *Corrupt*(INS_*SN*_^*i*^) to acquire the reserved information {*id*_*j*_, *x*_*N*__*j*_, *y*_*N*__*j*_, *ST*_*j*_, *Cha*_*j*_, *T*_*j*_} in *SN*_*j*_ and try to calculate Δ^*∗*^=*h*(*x*_*N*__*j*_^new*∗*^, *y*_*N*__*j*_^new*∗*^, *K*_*SH*_, *T*_2_) to testify the *K*_*SH*_'s correctness, where *x*_*N*__*j*_^new*∗*^=*μ* ⊕ *h*(*A*_2_, *MH*_*j*_, *T*_2_), *y*_*N*__*j*_^new*∗*^=*λ* ⊕ *h*(*T*_2_, *A*_2_, *MH*_*j*_), and *MH*_*j*_=*h*(*PUF*(Cha_*j*_)) ⊕ *ST*_*j*_. *A* has to break PUF to obtain *MH*_*j*_. The probability of breaking PUF is *Adv*_*A*_^PUF^. Therefore, we have
  (5) $$\begin{array}{c} \mathrm{Pr}\;\left[Success_{A}^{3}\right]-\mathrm{Pr}\;\left[Success_{A}^{2}\right]\leq Adv_{A}^{PUF}. \end{array}$$
Game_4_: which simulates *Execute* and *Send* queries are executed by *A* to launch the collision attacks. In line with the birthday paradox's definition, the possibility of a hash collision is *q*_*H*_^2^/2^*l*_*h*_+1^. Meanwhile, the collision probability of other transcripts is (*q*_*S*_+*q*_*E*_)^2^/2*n*. Hence, we have
  (6) $$\begin{array}{c} \mathrm{Pr}\;\left[Success_{A}^{4}\right]-\mathrm{Pr}\;\left[Success_{A}^{3}\right]\leq \frac{{\left(q_{S}+q_{E}\right)}^{2}}{2n}+\frac{q_{H}^{2}}{2^{l_{h}+1}}\text{.} \end{array}$$

The random bit *r* ∈ (0, 1), the probability of guessing *r* is 1/2, which is equal to guessing the session key. That is,

(7) $$\begin{array}{c} \begin{array}{c} \mathrm{Pr}\;\left[Success_{A}^{4}\right]=\frac{1}{2} \end{array}\text{.} \end{array}$$

Combining (1) with (6), we got

(8) $$\begin{array}{c} \frac{1}{2}Adv_{A}^{P}\leq \frac{{\left(q_{S}+q_{E}\right)}^{2}}{2n}+\frac{q_{H}^{2}}{2^{l_{h}+1}}+Adv_{A}^{CDHP}+Adv_{A}^{PUF}\text{.} \end{array}$$

(8) can be expressed as follows:

(9) $$\begin{array}{c} Adv_{A}^{P}\leq \frac{{\left(q_{S}+q_{E}\right)}^{2}}{n}+\frac{q_{H}^{2}}{2^{l_{h}}}+2Adv_{A}^{CDHP}+2Adv_{A}^{PUF}\text{.} \end{array}$$

## 7. Performance Analysis

We study and compare security and performance efficiency between ours with others. According to the comparison of the security attributes which are given in Table 2, we earn better security. In Windows 10 professional 64-bit, Intel(R) Core(TM) i5-4590, we earn *T*_*HS*_=0.068ms (millisecond), *T*_*EA*_=2.501ms, *T*_*SE*_=0.56ms [36], where *T*_*HS*_ is hash operation, *T*_*EA*_ represents ECC operation, and *T*_*SE*_ is symmetric key encryption. As Table 3 revealed, we describe the computational cost comparison between other protocols and the proposed protocol. In [14], the server's and sensor's total computation cost is 5T_HS_+3T_HS_=8T_HS_(0.544ms). Accordingly, the schemes [29, 30] both need 6T_HS_+4T_HS_=10T_HS_(0.544ms), and scheme [25] needs 5T_HS_+5T_EA_+3T_SE_(14.525ms), and ours is 18T_HS_+6T_EA_(16.230ms). Because our protocol is safer than others and achieves perfect forward secrecy, so ours achieve both high computational efficiency and security.

According to [38], outputs of identity, timestamp, and password are 32 bits, and a random integer, hash function, or block encryption is 256 bits, and a point in the elliptic curve is 160 bits. We calculate the storage overhead of the devices participating in authentication. Storage costs comparison is indicated in Table 4, ours maintain the lowest storage overhead. In addition, messages in login and mutual authentication are transmitted 4 times in our scheme. We calculate our communication costs and others, and ours is equivalent to other schemes from Table 5.

## 8. Conclusion

We first point out that Alzahrani et al.'s protocol can't defend against stolen-verifier attacks, desynchronization attacks, known-key attacks, and off-line identity guessing attacks and has no perfect forward secrecy. After that, we design a patient monitoring scheme based on ECC for WBAN in IoHT. We use verification tool ProVerif and formal security proof to demonstrate the security of our scheme. Through comparative analysis, our protocol is safer and more efficient to suit the lightweight and secrecy in medical scenarios. In the future, we will research more pragmatic and anonymous authentication protocol for more complex WBAN scenarios.

## Figures and Tables

**Figure 1:** System model.

**Figure 2:** Mutual authentication and key agreement phase.

**Figure 3:** Definitions.

**Figure 4:** Events.

**Figure 5:** Queries.

**Figure 6:** The process of the sensor node **SN**_**j**_.

**Figure 7:** The process of MS.

**Figure 8:** Main process.

**Figure 9:** Results.

**Table 1:** Notations.

Notations	Description
*SN*_*j*_	*j* ^th^ sensor node
*RN*	Relay node
*MS*	Medical server node
*SA*	Server administrator
*AR*	The adversary
*id*_*j*_, *id*_*R*_	Identity of *SN*_*j*_/identity of *RN*
*K*_*MS*_, *Q*	Secret key and public key of *MS*, where Q=K_*MS*_∙P
*K*_*SH*_	Session key
*r*, *P*_*R*1_, *P*_*R*2_	Random integers
*b*_*j*_	Random number generated by *SN*_*j*_
*m, r* ^new^	Random integers generated by *MS*
*a*_*j*_, *r*, *P*_*R*1_, *P*_*R*2_	Random integers generated by *SA*
*T*, *T*_1_, *T*_2_, *T*_3_, *T*_4_	Timestamps
*P*	The base point of the elliptic curve
⊕	XOR operation
PUF(∙)	Physically unclonable function
*h*(∙)	Hash function
Δ*T*	The maximum transmission delay

**Table 2:** Security properties comparison.

Attacks/Properties	[14]	[25]	[29]	[30]	Ours
Anonymity	Yes	Yes	No	No	Yes
Mutual authentication	Yes	Yes	Yes	Yes	Yes
Forger and impersonation attack	No	Yes	Yes	Yes	Yes
Off-line identity guessing attack	Yes	Yes	No	No	Yes
Sensor node capture attack	Yes	Yes	Yes	Yes	Yes
Smart card loss attack	Yes	Yes	Yes	Yes	Yes
Desynchronization attack	Yes	No	Yes	No	Yes
Stolen‐verifier attack	Yes	Yes	Yes	No	Yes
Man-in-middle attack	Yes	Yes	Yes	Yes	Yes
Replay attack	Yes	Yes	No	Yes	Yes
Know-key attack	Yes	Yes	No	No	Yes
Untraceability	Yes	Yes	Yes	Yes	Yes
Perfect forward secrecy	No	No	No	No	Yes

**Table 3:** The computation cost comparison.

Schemes	Server	*SN*_*j*_ (sensor)	Total
[14]	5*T*_*HS*_	3*T*_*HS*_	8*T*_*HS*_(0.544*ms*)
[25]	3*T*_*HS*_+3*T*_*EA*_+2*T*_*SE*_	2*T*_*HS*_+2*T*_*EA*_+*T*_*SE*_	5*T*_*HS*_+5*T*_*EA*_+3*T*_*SE*_(14.525*ms*)
[29]	6*T*_*HS*_	4*T*_*HS*_	10*T*_*HS*_(0.680*ms*)
[30]	6*T*_*HS*_	4*T*_*HS*_	10*T*_*HS*_(0.680*ms*)
Ours	5*T*_*HS*_+3*T*_*EA*_	13*T*_*HS*_+3*T*_*EA*_	18*T*_*HS*_+6*T*_*EA*_(16.230*ms*)

**Table 4:** The storage cost comparison.

Protocols		Storage cost (bits)	Total (bits)
[14]	Sensor	544	864
	RN	32	
	Server	288	
[25]	Sensor	1536	1952
	RN	0	
	Server	416	
[29]	Sensor	800	1108
	RN	32	
	Server	276	
[30]	Sensor	1056	1664
	RN	32	
	Server	576	
Ours	Sensor	832	928
	RN	32	
	Server	64	

**Table 5:** The communication cost comparison.

Schemes	[14]	[25]	[29]	[30]	Ours
Communication cost (bits)	4196	2752	3712	3712	3936

## Data Availability

All data are included in manuscript.
